The article "Screening and Identification of Antidepressant Active Ingredients from Puerariae Radix Extract and Study on Its Mechanism" was retracted in 2024. Reasons: signs of a paper mill; suspected computer-generated content; unreliable results or conclusions; concerns about the data.

# Screening and Identification of Antidepressant Active Ingredients from *Puerariae Radix* Extract and Study on Its Mechanism

**DOI:** 10.1155/2021/2230195

**Published:** 2021-09-09

**Authors:** Guoze Wang, Peng Luo, Shuai Zhang, Qun Huang, Shuling Zhang, Qibing Zeng, Jingxin Mao

**Affiliations:** ^1^School of Public Health, The Key Laboratory of Environmental Pollution Monitoring and Disease Control, Ministry of Education, Guizhou Medical University, Guiyang 550025, China; ^2^State Key Laboratory of Functions and Applications of Medicinal Plants, Guizhou Medical University, Guiyang 550014, China; ^3^Department of Interventional Radiology, The Affiliated Cancer Hospital of Guizhou Medical University, Guiyang 550000, China; ^4^College of Pharmaceutical Sciences, Southwest University, Chongqing 400715, China

## Abstract

*Objective*. Depression is a common mental disease with long course and high recurrence rate. Previous studies showed that *Puerariae Radix* and its extracts have powerful antidepressant effects in recent years. The study proposed an integrated strategy, combining network pharmacology and molecular pharmacology experiment to investigate the mechanisms of the antidepressant active ingredients from *Puerariae Radix. Methods*. TCMSP database, GeneCards database, Venny 2.1, UniProt database, STRING database, Cytoscape 3.7.2, and Metascape database were used to screen the active chemical components, antidepressant-related genes, and core targets, convert the abbreviated gene names in batch, search and predict the interaction between proteins, and construct the PPI network of *Puerariae Radix*. KEGG pathway and GO biological process enrichment and biological annotation were used to select antidepressant core gene targets. The MTT method was used to detect the effect of puerarin on the damage of PC12 cells induced by corticosterone. The DCFH-DA probe and ROS assay kit were utilized to detect the production of ROS in PC12 cells. PI/Annexin V was used to detect the apoptotic rate of puerarin on PC12 cells. Western blotting was used to verify the regulation of puerarin on the key targets of AKT1, FOS, CASP3, STAT3, and TNF-*α* in PC12 cells. *Results and Conclusion*. Eight main active components, 64 potential antidepressant gene targets, and 15 core antidepressant gene targets were obtained. 35 signaling pathways and 52 biological processes related to antidepressant effect of *Puerariae Radix* were identified. Puerarin was the active ingredient derived from *Puerariae Radix* which exhibited the antidepression effect by improving the viability of cell, reducing cell apoptosis, regulating ROS production, increasing protein expressions of AKT1 and FOS, and reducing protein expressions of CASP3, STAT3, and TNF-*α*. The study revealed the pharmacodynamic material basis and possible antidepressant mechanism of *Puerariae Radix* and provided new theoretical basis and ideas for antidepressant research.

The article "Screening and Identification of Antidepressant Active Ingredients from Puerariae Radix Extract and Study on Its Mechanism" was retracted in 2024. Reasons: signs of a paper mill; suspected computer-generated content; unreliable results or conclusions; concerns about the data.

## 1. Introduction

Depression is a severe affective mental disorder caused by various reasons such as violence, drug abuse, and psychological frustration, which is defined as a cluster of special symptoms with related disorders [1]. Due to major changes in physical, psychological, and social relationships, the incidence of depression has risen sharply [2], and statistics showed that the initial prevalence of depression is 3% to 8% [3]. At the same time, due to the longer course of depression and the higher recurrence rate, the lifetime probability of illness is as high as 11 to 20% [4], and its high morbidity and high suicide rate have also attracted more and more attention. At present, drug therapy is still one of the main means of treating depression, and most of the antidepressant drugs used in clinical are chemical drugs. Chemical antidepressants mainly include selective serotonin reuptake inhibitors (SSRIs) such as fluoxetine, paroxetine, and escitalopram; tricyclics (TCAs) such as chlorpromazine, doxepin, and amitriptyline; tetracyclics (TeCAs) such as sertraline, maprotiline, and mianserin; and monoamine oxidase inhibitors (MAOI) such as phenelzine, brofaromine, and tolosa ketone. However, long-term use of these drugs may cause adverse reactions, including the risk of causing serotonin syndrome, triggering autonomic dysfunction, having liver toxicity, and inducing cardiovascular disease [5].

Traditional Chinese Medicine (TCM) is rich in resources and has a complete theoretical system which has a history of thousands of years in clinical application, searching for natural medicines with clear curative effect, small toxic and side effects, and safety and high efficiency from TCM for antidepressant treatment which has broad prospects [6]. *Puerariae Radix* is the dry root of *Pueraria lobata* (Willd. Ohwi) or *Pueraria thomsonii* Benth which mainly produced in Guangdong, Hunan, Henan, and Zhejiang, China. An important TCM-related ancient book named “Treatise on febrile and miscellaneous diseases” has been recorded the significant effects of *Pueraria lobata* on relieving muscles, reducing fever, and rejuvenating and relieving diarrhea. In addition, “Gegen decoction,” a famous prescription, may develop the “Qi” on in the spleen and stomach. “Compendium of Materia Medica” also records that *Pueraria lobata* has coolness, calmness, and sweet taste with effects of clearing heat, reducing fire, and detoxifying. The 2015 edition of the “Pharmacopoeia of the People's Republic of China” has been recorded that *Pueraria lobata* can be used to treat fever, thirst, acute dysentery, diarrhea, diabetes, and hypertension [7]. Studies in the field of modern chemistry and medicine have shown that the main chemical constituents of *Pueraria lobata* include isoflavones, triterpenes, coumarins, and alkaloids [8]. It was reported that the extract of *Puerariae Radix* and its monomeric compounds have the effects on antioxidation [9], antihigh blood pressure [10], anticancer [11], antidiabetes/nephropathy [12], and neuroprotective [13].

The article "Screening and Identification of Antidepressant Active Ingredients from Puerariae Radix Extract and Study on Its Mechanism" was retracted in 2024. Reasons: signs of a paper mill; suspected computer-generated content; unreliable results or conclusions; concerns about the data.

In addition, previous studies have found that *Puerariae Radix* and its extracts have powerful antidepressant effects in recent years. It was reported that the ethanol extract of *Puerariae Radix* can significantly shorten the fixed time of the forced swimming test (FST) and tail suspension test (TST) with cerebral ischemia-reperfusion and reverse the norepinephrine (NE) and 4-dihydroxyphenylacetic acid-induced ptcerebral ischemia-reperfusion of protein in the hippocampus and striatum of mice [14]. It has been demonstrated that *Pueraria lobata* Ohwi could ameliorate depression-related behavior, including in FST and TST that are influencing depression in an ovariectomized rat menopause model [15]. It was revealed that the combination of *Puerariae Radix* and hawthorn fruit could prevent depression in a diabetic rat model [16]. It was found that the acute antidepressant effects of *Puerariae Radix* extract on poststroke depression mice further significantly increased the tyrosine hydroxylation of hippocampus enzyme mRNA expression through behavior and gene expression experiments [17]. It was also reported that *Puerariae Radix* as major constituents of Chaihu-Shugan-San which could obviously improve the depressive state of the model rats and its mechanism may be correlated with regulating the expressions of JNK in the hippocampus [18]. Furthermore, the monomer compounds which were extracted from *Puerariae Radix also* exhibit excellent antidepressant activity in recent research. It was revealed that after 14 days of continuous administration of isoflavone pueraria which extracted from *Puerariae Radix*, the fixed time of FST and TST was significantly shortened, and the serotonin-induced mouse convulsions/head flicking behavior was significantly enhanced in a dose-dependent manner. Puerarin isoflavones also have obvious antagonistic effects on resuscitation-induced eyelid atrophy, dyskinesia, and hypothermia [19].

Network pharmacology is developed based on system biology and computer technology, and it integrates the knowledge of bioinformatics and pharmacology, and through the construction of the “component-target-gene-disease” network, a comprehensive analysis of the drug on the human body influences, thus revealing the mechanism of action of multiple components and multiple targets on disease. In recent years, with the rapid development of bioinformatics, network pharmacology has played an important role in predicting and identifying effective ingredients, targets, related diseases, and pharmacological mechanisms of TCM. The chemical composition of TCM and its compounds are complex, with the synergy of multicomponent and multitarget, which have the advantages of holistic treatment, and can overcome the shortcomings of poor single-target western medicine.

The article "Screening and Identification of Antidepressant Active Ingredients from Puerariae Radix Extract and Study on Its Mechanism" was retracted in 2024. Reasons: signs of a paper mill; suspected computer-generated content; unreliable results or conclusions; concerns about the data.

Patients with depression often have intractable sleep disorders, with an incidence of up to 98%, which are manifested in insomnia, difficulty falling asleep, early awakening, sleep rhythm disorder, poor sleep quality with long course of disease, and high recurrence rate [20]. Previous studies have been demonstrated that *Puerariae Radix* and its extracts have powerful antidepressant effects in recent years [14–19]. However, because of the complex composition of *Puerariae Radix*, its main material basis and molecular mechanism for the treatment of depression are still unclear. Therefore, the pharmacodynamic material basis of *Puerariae Radix* and its possible antidepressant mechanism was studied through the network pharmacology method by screening of active ingredients, target prediction, PPI network construction, KEGG pathway, and GO biological process analysis.

Currently, the cells used for depression research and antidepressant drug screening include SH-SY5Y neuroblastoma cells [21], primary cultured cells (neural stem cells, microglia cells, and astroglia cells) [22–24], glioma C6 cells [25], and pheochromocytoma (PC12) cells [26]. Among them, cort-induced PC12 cells are the most widely used as the in vitro models of depression. Therefore, cort-induced PC12 cells were finally chosen for establishing the depression-like model. In the present study, molecular biology experiments were also used to verify the antidepressant active ingredients and mechanism of *Puerariae Radix* in PC12 cells, combining network pharmacology method and molecular pharmacology experiment to ascertain the active ingredients from *Puerariae Radix* and study on its antidepressant mechanism.

## 2. Materials and Methods

### 2.1. Applied Network Database and Software

The TCM pharmacology database and analysis platform (TCMSP, https://tcmspw.com/tcmsp.php/), GeneCards database (https://www.genecards.org/) UniProt, a general protein database (https://www.uniprot.org/), protein interaction platform STRING version 11.0 (https://string-db.org/), the biological information annotation database Metascape (https://metascape.org/gp/index.html#/main/step1), and network topology attribute analysis software Cytoscape 3.7.2 were used for analysis and plotting.

The article "Screening and Identification of Antidepressant Active Ingredients from Puerariae Radix Extract and Study on Its Mechanism" was retracted in 2024. Reasons: signs of a paper mill; suspected computer-generated content; unreliable results or conclusions; concerns about the data.

### 2.2. Screening of Active Components and Targets of *Puerariae Radix*

TCMSP is a systematic pharmacology database and analysis platform of TCM developed by Chinese research team, which integrates pharmacokinetics, pharmacochemistry, and drug target protein network disease network. It can be linked with the databases such as DrugBank, TTD, and HIT to obtain the target protein and disease information and finally form the “drug-target-disease” network for TCM. The active components and targets of *Puerariae Radix* were obtained by searching “*Puerariae Radix*” in application of the TCMSP database and analysis platform. Then, according to the standard of oral bioavailability (OB) ≥ 20%, the main active components and targets of *Puerariae Radix* were screened.

### 2.3. Construct the Target Network of Active Components of *Puerariae Radix*

The UniProt database was used to identify the active components and corresponding target proteins of *Puerariae Radix* from “1.2” and unified conversion to abbreviated gene names. Cytoscape is a free software for building, visualizing, and analyzing networks. The active components and their corresponding targets of *Puerariae Radix* were imported into Cytoscape 3.7.2. The network graph of “active components-targets of *Puerariae Radix*” was constructed, and the topological data such as degree value and betweenness were derived. The topological properties of *Puerariae Radix* were analyzed by using the function of “network analyzer.” Degree and betweenness are important topological parameters to evaluate the proportion of nodes in the network. Degree value can reflect the number of links between one node and other nodes, while the betweenness reflects the ratio of the number of paths passing through the node to the total number of shortest paths in the network. After the results are visualized and output, the active components and targets of *Puerariae Radix* were represented by nodes, and the interaction between the two nodes was represented by edges. The degree of a node is the number of edges connected to the node. The greater the degree, the more nodes in the network that are directly related to the node, indicating that the node is more important in the network.

### 2.4. Collection of Antidepression-Related Targets of *Puerariae Radix* Active Compounds

The GeneCards database is a platform that provides all known human genes in genome, proteome, transcription, genetics, and function. Using “antidepressant” as a keyword, search for target information related to depression in the GeneCards database. Using Venny 2.1, the target of antidepressant was mapped with the target of active ingredient of *Puerariae Radix*, and the common target was selected as the related target of antidepressant of active ingredient of *Puerariae Radix*. Then, it was imported into Cytoscape 3.7.2 to construct the target network of “active compound-antidepressant of *Puerariae Radix*,” and its topological properties were analyzed by using the “network analyzer” function.

The article "Screening and Identification of Antidepressant Active Ingredients from Puerariae Radix Extract and Study on Its Mechanism" was retracted in 2024. Reasons: signs of a paper mill; suspected computer-generated content; unreliable results or conclusions; concerns about the data.

### 2.5. Construction of Target Protein Interaction (PPI) Network

The STRING database is mainly used to search and predict the interaction between proteins. In order to study the interaction between the target proteins of *Puerariae Radix* active components in the treatment of depression, the PPI network of related target proteins was constructed using the STRING version 11.0 platform. The species (protein species) was set as “Homo sapiens” (human), and the minimum interaction threshold was set to “medium confidence” 0.7 with medium confidence, and the remaining parameters remained at the default settings. Then, the network analyzer function in the software of Cytoscape 3.7.2 is used to study the topological properties of the PPI network and draw the PPI network diagram.

### 2.6. Kyoto Encyclopedia of Genes and Genomes (KEGG) Pathway Analysis and Gene Function Annotation (GO) Bioaccumulation Analysis

Biological information annotation database Metascape integrates several authoritative data resources, such as UniProt, DrugBank, KEGG, and GO, which can provide comprehensive biological function annotation information. Compared with the DAVID database, which is slow to update data, Metascape includes the latest, most comprehensive, and significant enrichment effect of biological annotation. The KEGG pathway and GO biological process enrichment analysis of core genes which were obtained in 1.5 were carried out by the Metascape database. The key target genes were screened by setting the threshold *P* < 0.05 as the critical value of significant functions and pathways. The main pathways and biological processes with significant differences in antidepressant pharmacological effects of the main active components of *Puerariae Radix* were obtained.

### 2.7. Cell Experimental Verification In Vitro

Based on the preliminary analysis of network pharmacology, it was found that puerarin has a total of 55 gene targets for antidepressants and the strongest correlation with the depression signaling pathway. In addition, the drug similarity value (DL) of puerarin is 0.69, which is also the highest among all monomer compounds in *Puerariae Radix*. Based on this, in the follow-up molecular biology verification process, we selected puerarin, the single component with the most gene targets and the most potential for medicine, for follow-up experiments.

The article "Screening and Identification of Antidepressant Active Ingredients from Puerariae Radix Extract and Study on Its Mechanism" was retracted in 2024. Reasons: signs of a paper mill; suspected computer-generated content; unreliable results or conclusions; concerns about the data.

#### 2.7.1. Cell Lines and Drugs

The PC12 cell line was purchased from the Shanghai Cell Bank of the Chinese Academy of Sciences. Corticosterone was purchased from Sigma Co., Ltd. The entire plant of *Puerariae Radix* was collected from Dianjiang, Chongqing Province, and identified by professor Min Chen at College of Pharmaceutical Sciences, Southwest University. Puerarin was extracted from the ethyl acetate part of *Puerariae Radix* and refined into medicinal material with a purity > 99%. The primary extraction, isolation, and purification of puerarin showed as the following: powder of the air-dried roots (2 kg) of *Puerariae Radix* was extracted by maceration with 95% ethanol overnight at room temperature. The ethanol extract was evaporated in vacuo to yield a semisolid (0.23 kg), which was suspended in water (5 L) and partitioned with petroleum ether (15 L), ethyl acetate (15 L), and n-butanol (15 L), successively. The ethyl acetate solution was concentrated to yield 152 g of residue, which was subjected to silica gel chromatography and eluted with petroleum ether ethyl acetate mixtures of increasing polarity (99 : 1 to 10 : 1) to obtain total 16 fractions. Puerarin was obtained from fraction 5 (Fr. 5, 5.23 g) which was separated continuously to finally obtain puerarin (15.67 mg).

#### 2.7.2. Main Instruments

The main instruments are Model 311 CO_2_ cell incubator (Thermo Fisher Scientific), HH-6 digital display constant temperature water bath (Jiangsu Jintan Ronghua Instrument Manufacturing Co., Ltd.), LDZX-30KBS vertical sterilizer (Shanghai Shen'an Medical Equipment Factory), 680 microplate reader (Bio-Rad), TG16-WS high-speed centrifuge (Shanghai Hu Yueming Scientific Instrument Co., Ltd.), BDS inverted microscope (Auto Optics), 24DN electrophoresis apparatus (Beijing Liuyi Instrument Factory), TS-2000A Shaker (Jiangsu Haimen Qilin Bell Instrument Manufacturing Co., Ltd.), DYCZ-40D Film Transfer Instrument (Beijing Liuyi Instrument Factory), Purelab classic series water purifier (Elga company), and ChemiDoc™ Touch Imaging System chemiluminescence imaging system (Bio-Rad company).

#### 2.7.3. Main Reagents

The main reagents are RPMI-1640 medium (Invitrogen company), fetal bovine serum (Thermo Fisher Scientific company), trypsin (Thermo Fisher Scientific company), ultrapure water (Elga company), penicillin/streptomycin (Biyuntian Institute of Biotechnology), MTT kit (Nanjing Jiancheng Institute of Biological Engineering), cell lysate, BCA protein concentration determination kit (Nanjing KGI Biotech Co., Ltd.), prestained protein Marker (Nanjing Kai solution (Tris-Glycine Transfer Buffer), Tris-glycine protein) Electrophoresis solution (T-based biological company), PVDF membrane, ECL luminescence kit (Beijing Baierdi Biotechnology Co., Ltd.), primary antibody: TNF-*α*, AKT1, FOS, STAT3, CASP3 (Abcam company), secondary antibody: goat anti-rabbit IgG, and GAPDH as an internal reference gene (Cell Signaling Technology). Protein lysis buffer, polyacrylamide gel electrophoresis gel preparation kit, Tris-glycine transfer buffer (Tris-Glycine SDS Buffer), polyacrylamide gel Electrophoresis protein loading buffer (SDS-PCAGE Loading Buffer), PBS, and TBST were purchased from Beijing Kangwei Century Biotechnology Co., Ltd.

The article "Screening and Identification of Antidepressant Active Ingredients from Puerariae Radix Extract and Study on Its Mechanism" was retracted in 2024. Reasons: signs of a paper mill; suspected computer-generated content; unreliable results or conclusions; concerns about the data.

#### 2.7.4. Cell Culture

PC12 cells were placed in a 6-well culture dish and cultured in RPMI-1640 medium, 10% fetal bovine serum, and 1% penicillin/streptomycin in a 37°C, 5% CO_2_ incubator. The medium was changed every day. After three days, PC12 cells were digested by trypsin and passaged. While passaged for three times, they were inoculated into 6-well plates at a density of 1 × 10^5^ cells/mL.

#### 2.7.5. MTT Method to Detect Corticosterone Toxicity

PC12 cells were taken in the logarithmic growth phase and inoculate them in a 48-well plate and adjust the final concentration to 1 × 10^5^/mL. Place them in a 37°C, 5% CO_2_ incubator for 48 hours, discard the supernatant, and add 100, 200, and 400 *μ*mol/L corticosterone, respectively, with 3 replicate holes in each group. After 24 hours of incubation, 10 *μ*L of MTT (5 mg/mL) was added to each well and then incubated for another 4 hours. The optical density (OD) of absorbance was measured at 450 nm.

#### 2.7.6. Detection of PC12 Cell Viability by MTT Method

After inoculating PC12 cells in the logarithmic growth phase in a 96-well plate, place them in a 5% CO_2_ incubator and incubate for 24 hours. 20 *μ*L of MTT (5 mg/mL) solution was added to all experimental setup groups and continued to incubate for 4 hours with PBS, then washed 3 times, and discarded the culture medium, and 100 *μ*L DMSO was added to each well and shaked at low speed for 10 minutes to fully dissolve the crystals. The experiment includes control group, corticosterone (model) group, low-concentration puerarin group (50 *μ*mol/L puerarin), medium-concentration puerarin group (100 *μ*mol/L puerarin), and high-concentration puerarin group (150 *μ*mol/L puerarin), and each group was treated with 100 *μ*L of 200 *μ*mol/L corticosterone, respectively, for 24 hours except for the control group and then treated with different concentrations of puerarin for 24 hours. Finally, 10 *μ*L of MTT was added to each well, cultured for 4 hours, and then, the OD value was measured at 450 nm.

The article "Screening and Identification of Antidepressant Active Ingredients from Puerariae Radix Extract and Study on Its Mechanism" was retracted in 2024. Reasons: signs of a paper mill; suspected computer-generated content; unreliable results or conclusions; concerns about the data.

#### 2.7.7. Detection of the ROS Level in PC12 Cells

The logarithmic growth phase of PC12 cells was incubated with DMEM medium containing 10% fetal bovine serum in 96-well culture plates with cell concentration of 1 × 10^5^ pcs/mL for 12 hours. Cells were divided into control group, model group, 50 *μ*mol/L puerarin group, 100 *μ*mol/L puerarin group, and 150 *μ*mol/L puerarin group. PC12 cells were spread on a 6-well plate and divided into 6 groups. Set three parallel tubes in each group and repeat three times independently. Perform experiments in strict accordance with the kit instructions.

Reactive oxygen species (ROS) level was detected by ROS assay kit. PC12 cells in logarithmic growth phase were inoculated into 48-well plates and divided into 5 groups including control group, model group, 50 *μ*mol/L puerarin group, 100 *μ*mol/L puerarin group, and 150 *μ*mol/L puerarin group. Each group was provided with three multiple pores, and the final concentration of 10 *μ*M DCFH-DA was incubated in 37°C incubator for 30 minutes. After incubation, cells were washed with PBS. The fluorescence microscope was used to observe and capture the image, and the fluorescence intensity was analyzed by the Image-Pro Plus software.

#### 2.7.8. PI/Annexin V Detects PC12 Cell Apoptosis Rate

The PC12 cells in the logarithmic growth phase were digested and centrifuged and then resuspended in the culture medium. Adjust the cell density to 1 × 10^5^ cells/mL and culture the cells in a 5% CO_2_ incubator overnight. The adherent cells were cultured in different concentrations (50, 100, and 150 *μ*mol/L) of puerarin for 48 hours and then digested, washed, and collected on a 48-well culture plate. According to the instructions of the apoptosis kit, add 500 *μ*L buffer to each well to resuspend the cells, then add 5 *μ*L each of PI and Annexin to each well, incubate for 15 minutes in the dark, and finally use a flow cytometer to detect the rate of apoptosis.

#### 2.7.9. Detection of the Expression of Key Proteins in Depression-Related Signaling Pathways

Add 300 *μ*L of cell lysate, lyse on ice for 30 minutes, then scrape the cells with a cell scraper, add them to a blank EP tube, use a centrifuge at 12000 r/min, take the supernatant, and add protein loading buffer at a ratio of 4 : 1, 100°C or boiling water bath for 3~5 minutes to fully denature the protein. The protein samples were separated with 12.5% SDS-PAGE and transferred onto PVDF membranes. The membrane was washed 3 times with TBST, and each time is 10 minutes. Blots were blocked in 10% skim milk at room temperature for 1 hour and incubated overnight at 4°C with primary antibodies: AKT1 (1 : 1000), FOS (1 : 1000), STAT3 (1 : 1000), CASP3 (1 : 1000), and TNF-*α* (1 : 1000). Take out the washing membrane the next day and incubate it in the secondary antibody (1 : 1000) for 1 hour. According to the molecular weight, select the range of rubber cutting, using the ECL luminescence method to develop; the experiment is repeated three times, and the gray value of the band is calculated and analyzed.

The article "Screening and Identification of Antidepressant Active Ingredients from Puerariae Radix Extract and Study on Its Mechanism" was retracted in 2024. Reasons: signs of a paper mill; suspected computer-generated content; unreliable results or conclusions; concerns about the data.

#### 2.7.10. Statistical Analysis

The SPSS 19.0 software and the ImageJ software were used to perform statistical processing and gray value analysis on the experimental data, respectively. The GraphPad Prism 8 software was used to make graphs. The one-way analysis of variance (ANOVA) method was used for statistical analysis, and *P* < 0.05 (5% significance level) and *P* < 0.01 (1% significance level) indicated that the difference was statistically significant.

## 3. Results

### 3.1. Screening Results of Main Active Chemical Components in *Puerariae Radix*

Screening for the values of OB ≥ 20% in the TCMSP database, a total of 8 active components of *Puerariae Radix* were finally obtained. They were formononetin, sitogluside, *β*-sitosterol, 3′-methoxydaidzein, (R)-allantoin, daidzein-4′, daidzein-4,7-diglucoside, puerarin, and 7,8,4′-trihydroxyisoflavone, respectively (Table 1).

### 3.2. *Puerariae Radix* Active Compounds Correspond to Potential Gene Targets

After searching through the TCMSP database and collecting the information on the gene targets, a total of 186 potential gene targets corresponding to the 8 active compounds of *Puerariae Radix* were collected (duplicates were not eliminated). Among them, formononetin contains 39 gene targets, sitogluside contains 17 gene targets, *β*-sitosterol contains 38 gene targets, and 3′-methoxydaidzein contains 19 gene targets. (R)-allantoin contains 2 gene targets, daidzein-4′,7-diglucoside contains 1 gene target, puerarin contains 55 gene targets, and 7,8,4′-trihydroxyisoflavone contains 15 gene targets. After eliminating the duplicates, a total of 99 targets corresponding to the active ingredients of *Puerariae Radix* were obtained, and a “compound-gene target network” was constructed using the Cytoscape 3.7.2 software (Figure 1(a), pink nodes represent drugs, and blue nodes represent gene targets). The overall situation of the distribution of the average degree value of each node in the network graph and the distribution of the betweenness centrality are shown in Figures 1(b) and 1(c).

The article "Screening and Identification of Antidepressant Active Ingredients from Puerariae Radix Extract and Study on Its Mechanism" was retracted in 2024. Reasons: signs of a paper mill; suspected computer-generated content; unreliable results or conclusions; concerns about the data.

### 3.3. *Puerariae Radix* Active Ingredient-Antidepression Target Network

Using the GeneCards database, searching “antidepressant” as a keyword, a total of 1,596 targets related to antidepressant were extracted. The gene targets corresponding to the active compounds obtained in the TCMSP database and the antidepression-related gene targets obtained from the GeneCards database were mapped to each other. Venn diagram was produced by the Venny 2.1 software, and finally, 64 common targets (3.9%) were obtained (Figure 2 and Table 2). The data were imported into Cytoscape 3.7.2 to construct the target network of “active compound-antidepressant” of *Puerariae Radix* (Figure 3(a), yellow nodes represent drugs, and blue nodes represent gene targets). The overall results of the average degree distribution and the betweenness centrality distribution of each node in the network diagram are shown in Figures 3(b) and 3(c).

### 3.4. Gene Target PPI Analysis

The data of antidepressant targets of *Puerariae Radix* in 2.3 were imported into the STRING database (version 11.0) to construct the PPI network of gene targets. Then, import the PPI network data into the software of Cytoscape 3.7.2 for visual analysis (Figure 4(a)), set the threshold value of degree > 15, and select 15 core targets according to the degree value from high to low (Table 3). These core targets were AKT1, FOS, CASP3, JUN, VEGFA, STAT3, PTGS2, MAPK14, ESR1, SIRT1, HSP90AA1, ACHE, SOD1, HIF1A, and AR. These target proteins are associated with depression, atherosclerosis, bipolar disorder, schizophrenia, Alzheimer's disease, insulin resistance, type 2 diabetes, and other diseases. In the present study, these core targets were visualized and analyzed by the Cytoscape 3.7.2 software (Figure 4(b)). The complete PPI network of antidepressant-related target proteins of *Puerariae Radix* was obtained finally.

### 3.5. KEGG Pathway Enrichment and GO Biological Process Analysis

KEGG pathway and GO analysis annotation were carried out for 15 core gene targets. Pathways were screened according to the principle of *P* < 0.05, and the top 20 KEGG pathways were listed according to the order of *P* value (Figure 5(a)). It mainly involves the regulation of ROS metabolism, the positive regulation of vascular endothelial cell migration, the regulation of aging, the regulation of neuron death, cytokine-mediated signaling pathway, the regulation of DNA binding transcription factor activity, toxic substance response, AGE-RAGE signaling pathway in diabetic complications, androgen receptor (AR) signaling pathway, hypoxia inducible factor (HIF) signaling pathway, and so on. The regulation of neuronal death, aging, reactive oxygen species metabolism, cytokine-mediated signaling pathway, and androgen receptor signaling pathway are closely related to depression.

The article "Screening and Identification of Antidepressant Active Ingredients from Puerariae Radix Extract and Study on Its Mechanism" was retracted in 2024. Reasons: signs of a paper mill; suspected computer-generated content; unreliable results or conclusions; concerns about the data.

The significance of GO biological process and molecular function enrichment of 15 core gene targets are also strictly screened according to the principle of *P* < 0.05. The analysis results of the top 20 are shown in Figure 5(b). These targets are related to a variety of biological processes, including biological adhesion, tissue cell composition or biogenesis, behavior, negative regulation of biological process, multicellular organic process, positive regulation of biological process, response to stimulation, biological regulation, immune system process, cell proliferation, and cell process. The occurrence of depression involves many abnormal biological processes in the body, which are closely related to the occurrence and development of depression. In addition, it was also suggested that *Puerariae Radix* may exhibit antidepressant effects by regulating these biological processes.

### 3.6. Effect of Corticosterone on the Activity of PC12 Cells

Compared with the control group, the activity of PC12 cells treated with different concentrations of corticosterone was significantly reduced, and there was a statistically significant difference (*P* < 0.01), which indicates that the model was successfully established (Figure 6(a)). In addition, while the concentration of corticosterone was 200 *μ*mol/L, the survival rate of PC12 cells was between 40 and 50%, which might better clarify the difference between PC12 cell damage and protective factors. Therefore, 200 *μ*mol/L corticosterone was selected as the appropriate model concentration for follow-up research.

### 3.7. Effect of Puerarin on the Activity of Corticosterone-Induced Injury of PC12 Cells

Compared with the control group, the PC12 cell viability of the corticosterone group was significantly reduced (*P* < 0.01); compared with the model group, the PC12 cell viability of the medium and high concentrations of the puerarin group was significantly enhanced (*P* < 0.05 and *P* < 0.01), and the medium and high concentration of puerarin can significantly improve the viability of damaged PC12 cells induced by corticosterone at a concentration of 200 *μ*mol/L (Figure 6(b)).

### 3.8. Effect of Puerarin on Corticosterone-Induced ROS Generation in PC12 Cells

Although the pathogenesis is different, oxidative stress is a common factor in the occurrence and development in nervous system diseases. Previous studies have shown that a large number of ROS might be produced in the nerve cells of specific brain regions due to different reasons of injury [27]. In order to study whether corticosterone induced ROS production in PC12 cells, the expression level of ROS in corticosterone-treated L-02 cells was evaluated by detecting the oxidative transformation from nonfluorescent DCFH-DA to fluorescent DCF. Compared with the control group (Figure 7(a)), it was shown that corticosterone triggered ROS production in PC12 cells (Figure 7(b)). Compared with the control group, the ROS production in PC12 cells was significantly increased after intervention with corticosterone (600 mM) for 8 h. Compared with the model group, pretreatment with different concentrations of puerarin can significantly inhibit the production of ROS in PC12 cells induced by corticosterone (Figures 7(c)–7(e)). It was revealed that the production of ROS was significantly reversed with the increase of puerarin concentration.

The article "Screening and Identification of Antidepressant Active Ingredients from Puerariae Radix Extract and Study on Its Mechanism" was retracted in 2024. Reasons: signs of a paper mill; suspected computer-generated content; unreliable results or conclusions; concerns about the data.

### 3.9. Effect of Puerarin on Corticosterone-Induced PC12 Cell Apoptosis

The results of the apoptosis rate of PC12 cells are shown in Figure 8. After treating PC12 cells with different concentrations of puerarin, they were labeled with PI/AnnexinV double staining and then detected by flow cytometry. Compared with the control group, the corticosterone group can significantly increase the apoptosis rate of PC12 cells (*P* < 0.01); compared with the corticosterone group, the different concentrations of the puerarin group can reduce the apoptosis rate of PC12 cells from 52.25% to 15.05%.

### 3.10. Effect of Puerarin on Protein Expression in Depression-Related Pathways

Compared with the control group, the expressions of AKT1 and FOS protein significantly decreased, while the expressions of CASP3, STAT3, and TNF-*α* protein significantly increased in the model group. Compared with the model group, the expressions of AKT1 and FOS protein were significantly increased (*P* < 0.01), and the expressions of CASP3 (*P* < 0.01), STAT3 (*P* < 0.05), and TNF-*α* (*P* < 0.05) protein were significantly reduced in the 50 *μ*mol/L puerarin group. The expressions of AKT1 and FOS protein were also significantly increased (*P* < 0.01) while the protein expressions of CASP3 (*P* < 0.01) and TNF-*α* (*P* < 0.01) were significantly decreased, and the protein expression of STAT3 has no significant change in the 100 *μ*mol/L puerarin group. The protein expressions of AKT1 and FOS protein were significantly increased (*P* < 0.01), while the expressions of CASP3, STAT3, and TNF-*α* protein were significantly reduced (*P* < 0.01) in the 150 *μ*mol/L puerarin group (Figure 9). The results confirmed the correctness of screening the active ingredient puerarin of *Puerariae Radix* in the treatment of depression through systematic network pharmacology.

## 4. Discussion

Nowadays, most studies are based on traditional pharmacological methods but not the methods of network pharmacology. Although traditional pharmacological methods can reveal the pharmacology and mechanism of drugs, these research methods are difficult to fully describe the complex relationship and molecular mechanism between drugs and the human body. In addition, a single chemical drug acting body belongs to a single target, which lacks the advantages of the overall argument compared with the synergistic effect of multicomponent and multitarget of TCM. Based on the development of system biology and multidirectional pharmacology, network pharmacology uses the network to integrate the biological network and the role of drugs, analyzes the relationship between drugs and nodes or network modules in the network, and uses multicomponent, multitarget, and multipathway mode of action. In the present study, 8 active chemical components such as formononetin, puerarin, and 7,8,4′-trihydroxyisoflavone and 99 potential gene targets were screened from the TCMSP database using network pharmacology methods. A total of 1,596 gene targets related to depression were searched in the GeneCards database. Using Venny 2.1, the obtained antidepression targets were mapped to the *Puerariae Radix* active ingredient targets and 64 common targets were selected. Then, the UniProt database was utilized to convert abbreviated gene names in batch, and the STRING database was used to search/predict protein interactions and construct a PPI network, and the Metascape database was used to enrich the selected antidepressant core genes by KEGG pathway and GO biological process enrichment analysis and biological notes; the Cytoscape 3.7.2 software for the PPI network was carried out to study topological properties, drawing the PPI network diagram. The material basis and molecular mechanism of antidepressant effect of *Puerariae Radix* were preliminarily analyzed.

The article "Screening and Identification of Antidepressant Active Ingredients from Puerariae Radix Extract and Study on Its Mechanism" was retracted in 2024. Reasons: signs of a paper mill; suspected computer-generated content; unreliable results or conclusions; concerns about the data.

Isoflavone is one of the flavonoids, mainly found in leguminous plant, which affect hormone secretion, metabolic biological activity, protein synthesis, growth factor activity, and so on. Previous studies have found that isoflavones have protective effects on hippocampal neurons, which may save cognitive deficits, improve learning and memory abilities, and enhance hippocampal neurogenesis to combat cognitive menopause and other symptoms, with multiple pharmacological activity [28]. NMR combined with mathematical modeling to calculate the nonnuclear chemical shifts of the antidepressant shielding and deshielding Bq motion points in the space to predict the antidepressant activity of the isoflavone compound formononetin in *Puerariae Radix*. It was found that the asymmetry (*η*) and tilt (*κ*) parameters of the heterocyclic center of the compound fluctuate within a small range and are optional at large distances. The calculated results indicate that the compound formononetin from *Puerariae Radix* has a significant antidepressant effect [29]. The pharmacological effects of formononetin on N-methyl-D-aspartic acid-induced neurotoxicity of primary cultured cortical neurons were studied. The results showed that 12-hour pretreatment of formononetin can significantly reduce the damage of N-methyl-D-aspartic acid to the cells and significantly reduce the number of apoptotic cells. The BCL2 and procaspase-3 levels were increased, and BAX and caspase-3 levels were reduced which regulates the expression of apoptosis-related proteins. It was indicated that formononetin has a neuroprotective effect and has potential application prospects for clinical treatment of degenerative diseases of the central nervous system [30]. It was also reported that formononetin may significantly increase the activity of glutathione peroxidase (GSH-Px) and superoxide dismutase (SOD) in brain tissue of rats with cerebral ischemia and reduce the malondialdehyde in the brain. The levels of malondialdehyde (MDA), tumor necrosis factor alpha (TNF-*α*), and interleukin 6 (IL-6) proved that formononetin mediated nerve cell damage, and its potential mechanism is related to the inhibition of inflammatory response in the brain and related to oxidative stress [31]. It has demonstrated that puerarin (60 mg/kg and 120 mg/kg) could reverse the distribution of progesterone, 5-hydroxytryptamine (5-HT), and 5-hydroxyindoleacetic acid (5-HIAA) in the prefrontal cortex and hippocampus of rats after long-term administration of isoflavone compounds (60 mg/kg and 120 mg/kg) and improve the behavior disorder caused by chronic stress in rats [32]. In addition, it was reported that puerarin treatment can effectively reduce chronic stress-induced depression (mainly hyposexuality and desperate behaviors) and may participate in the activation of hippocampal FGF-2 signal transduction and cellular responses, increasing the expression of FGF-2 [33]. It was found that the effects of puerarin on depression-like behavior and neuropathic pain in C57BL mice with nerve injury (SNI) can restore the consumption of reduced glutathione (GSH) and superoxide dismutase (SOD) induced by SNI and induce the expression of brain-derived neurotrophic factor (BDNF) rapidly and continuously thus effectively reducing depression and chronic pain in SNI mice [34].

PPI network analysis and screened out 15 core antidepressant targets were AKT1, FOS, CASP3, JUN, VEGFA, STAT3, PTGS2, MAPK14, ESR1, SIRT1, HSP90AA1, ACHE, SOD1, HIF1A, and AR. These target proteins are associated with depression, atherosclerosis, bipolar disorder, schizophrenia, Alzheimer's disease, insulin resistance, type 2 diabetes, and other disorders. Previous studies showed that protein kinase AKT1 may be related to the pathogenesis of affective disorders. It was reported that the AKT1 gene polymorphism rs1130214 is associated with antidepressant treatment response in patients with depression [35]. As a kind of nuclear protein transcription factor, FOS protein also plays an important role in regulating cell growth, division, proliferation, differentiation, and programmed death. Under normal circumstances, the c-fos gene participates in a variety of neuron activities, the expression of c-fos mRNA is very small, and the number of FOS-positive neurons is proportional to the stimulation intensity to a certain extent. Therefore, the expression of c-fos can be considered as a signal that nerve cells are activated by harmful stimuli. Whether long-term depression requires the transcription factor c-fos was studied which results showed that the application of c-fos in the brain prevented the occurrence of long-term depression, inhibited the increase of c-fos caused by long-term depression, and impaired spatial learning [36]. Vascular endothelial growth factor (VEGF) is one of the factors which play a role in the etiology and development of recurrent depression. Enzyme-linked immunoassay (ELISA) was used to measure circulating serum VEGF levels in 268 patients with recurrent depression and 200 Caucasians. The results showed that the VEGFA C allele and CC genotype were risk factors for recurrent depression. VEGFA mRNA expression and VEGF levels in patients with recurrent depression are higher than those in the control group; thus, VEGFA gene polymorphism can be used as a prognostic factor for the development of recurrent depression [37]. Neuron-microglia interaction plays a vital role in maintaining the nervous immune system, and the balance of the nervous immune system has become an important process in the pathophysiology of depression. Microglia-specific signal transducers and transcriptional activator 3 (STAT3) knockout mice were used to study microglial-derived synaptic changes to induce antidepressant-like behavior. The results showed that microglia-specific STAT3 knockout mice showed antidepressant-like behavior in forced swimming, tail suspension, sucrose preference, and field trials [38].

The article "Screening and Identification of Antidepressant Active Ingredients from Puerariae Radix Extract and Study on Its Mechanism" was retracted in 2024. Reasons: signs of a paper mill; suspected computer-generated content; unreliable results or conclusions; concerns about the data.

In order to further explore the biological pathways of antidepressant regulated by the active ingredients of *Puerariae Radix*, KEGG pathway enrichment and GO biological process analysis on the proteins were performed in the present study for the PPI network. It was found that the key targets of the PPI network and depression are closely related to interleukin (IL) signaling pathway, VEGFR1 signaling pathway, AR signaling pathway, HIF signaling pathway, cytokine-mediated signaling pathway, and other signaling pathways. The effects of stress on mouse behavior and cytokine expression activity were analyzed which results showed that mice under reduced stress experienced reduced sucrose consumption (indicating anaerobic behavior), increased climbing activity in the forced swimming test (indicating anxiety), and increased proinflammatory cytokine IL-6. The expression of anti-inflammatory cytokine IL-10 is reduced, and the results show that the IL signaling pathway is activated and participates in the biological behavioral effects of stress in mice [39]. VEGF is a vascular growth factor and permeability regulator, which is involved in the physiological and pathological processes of angiogenesis and the development of lymphatic vessels. VEGF produces biological effects by interacting with three VEGF receptor subtypes (VEGFR1, VEGFR2, and VEGFR3), where VEGFR1 signal transduction is very important for the cellular and behavioral responses of antidepressant drugs. Previous studies have shown that VEGF has neurotrophic and neuroprotective potential in the peripheral and central nervous system, and antidepressants can induce the expression of vascular endothelial growth factor in the hippocampus. HIF-1 is a transcriptional activator of VEGF, which can activate the cell's response to hypoxia [40]. HIF-1 is widely expressed in all cells, including peripheral leukocytes. The role of HIF-1 in depression and bipolar disorder was studied indicating that the expression levels of HIF-1*α* and HIF-1*β* mRNA in patients with depression and bipolar disorder were significantly higher than those in the healthy control group. Furthermore, it has demonstrated that the changes in the expression of HIF and its target genes may be related to the pathophysiology of depression [41].

The biological symptoms of depression include sleep disorders, appetite disorders, sexual dysfunction, energy loss, and some nonspecific physical symptoms, such as pain, general malaise, and autonomic dysfunction. Through analysis of GO biological processes of gene targets, we found that depression is associated with biological processes such as biological adhesion, response to stimuli, biological regulation, immune system processes, positive/negative biological processes, and cell proliferation. Epidemiological evidence indicates that there are irregular steady-state biological pathways in patients with depression, such as increased inflammation and disturbance of energy-regulated neuroendocrine signals (such as leptin and insulin) [42]. These changes in biological pathways indicate the relationship between depression and metabolic status (such as obesity, metabolic syndrome, and diabetes). Therefore, it is very important to study the above biological processes that are related to depression.

The article "Screening and Identification of Antidepressant Active Ingredients from Puerariae Radix Extract and Study on Its Mechanism" was retracted in 2024. Reasons: signs of a paper mill; suspected computer-generated content; unreliable results or conclusions; concerns about the data.

Scholars from various countries have found that puerarin can effectively reduce the occurrence and development of depression and reverse the behavioral disorders caused by chronic stress [32–34]. In addition, based on the preliminary analysis of network pharmacology, it was found that puerarin has 55 gene targets for antidepressant disease, and it is the monomer compound in pueraria that has the strongest correlation with depression signaling pathway. The drug similarity value (DL) of puerarin is 0.69, which is also the highest among all monomer compounds in *Puerariae Radix*. Therefore, in the follow-up molecular biology verification process, puerarin was finally selected as the active component with the most antidepressant gene targets and the most possible drug-making potential in *Puerariae Radix*, for follow-up experiments. The results showed that puerarin may significantly improve the viability of damaged PC12 cells induced by corticosterone at a concentration of 400 *μ*mol/L; significantly reduced the apoptotic rate of damaged PC12 cells induced by corticosterone; significantly decreased the production of ROS; significantly increased the protein expressions of AKT1 and FOS; and significantly reduced the protein expressions level of CASP3, STAT3, and TNF-*α*. The experimental results confirmed the accuracy of screening the active ingredient puerarin from *Puerariae Radix* in the treatment of depression-related targets through network pharmacology.

## 5. Conclusion

In conclusion, the present study firstly proposed an integrated strategy, combining molecular pharmacology experiment and network pharmacology to investigate the mechanisms of the antidepressant active ingredients from *Puerariae Radix.* A depression-like PC12 cell model was successfully established. The results of the present study suggest that puerarin which is derived from *Puerariae Radix* is the putative and active ingredient against depression. It significantly improved the viability of PC12 cells injured by corticosterone, reduced the apoptosis rate of PC12 cells injured by corticosterone, and decreased the production of ROS which induced by corticosterone. And it acted through the AKT1-STAT3 pathway by increasing protein expressions of AKT1 and FOS and reducing protein expressions of CASP3, STAT3, and TNF-*α* that are related to depression signaling pathways. Furthermore, the research will be required to investigate the optimum dose of puerarin and in vivo effect in the next step. Our study revealed the pharmacodynamic material basis and possible antidepressant mechanism of *Puerariae Radix* and provided new ideas for the systematic study of antidepressants at the cellular and molecular level.

The article "Screening and Identification of Antidepressant Active Ingredients from Puerariae Radix Extract and Study on Its Mechanism" was retracted in 2024. Reasons: signs of a paper mill; suspected computer-generated content; unreliable results or conclusions; concerns about the data.

## Figures and Tables

**Figure 1:** Active components of *Puerariae Radix*-prediction target network diagram and distribution map of degree value and betweenness centrality.

**Figure 2:** Venn diagram of common targets.

**Figure 3:** Active components of *Puerariae Radix-*antidepressant target network and distribution map of degree value and betweenness centrality.

**Figure 4:** PPI network of active compounds-antidepressant target protein of *Puerariae Radix.*

**Figure 5:** Enrichment analysis diagrams of KEGG pathway and GO biological process.

**Figure 6:** Effect of corticosterone and puerarin, respectively, on the activity of PC12 cells.

**Figure 7:** Effect of puerarin on corticosterone-induced ROS generation in PC12 cells.

**Figure 8:** Effect of puerarin on apoptosis of PC12 cells induced by corticosterone.

**Figure 9:** Effect of puerarin on protein expression in depression-related pathway.

**Table 1:** Easily absorbed active components and their basic parameters in *Puerariae Radix*.

ID	Ingredient	MW	AlogP	Hdon	Hacc	OB (%)	DL
MOL000392	Formononetin	268.28	2.58	1	4	69.67	0.21
MOL000357	Sitogluside	576.95	6.34	4	6	20.63	0.62
MOL000358	Beta-sitosterol	414.79	8.08	1	1	36.91	0.75
MOL002347	(R)-allantoin	158.14	-1.76	5	7	96.9	0.03
MOL002959	3′-Methoxydaidzein	284.28	2.32	2	5	48.57	0.24
MOL003629	Daidzein-4,7-diglucoside	578.57	-1.48	8	14	47.27	0.67
MOL012297	Puerarin	416.41	-0.06	6	9	24.03	0.69
MOL004631	7,8,4′-Trihydroxyisoflavone	270.25	2.07	3	5	20.67	0.22

**Table 2:** Antidepressant targets of active components from *Puerariae Radix.*

Gene	Target name
NOS2	Nitric oxide synthase 2
CHRM1	Cholinergic receptor muscarinic 1
ESR1	Estrogen receptor 1
AR	Androgen receptor
PTGS2	Prostaglandin-endoperoxide synthase 2
PDE3A	Phosphodiesterase 3A
ADRA1D	Adrenoceptor alpha 1D
SLC6A3	Solute carrier family 6 member 3
ADRB2	Adrenoceptor beta 2
SLC6A4	Solute carrier family 6 member 4
ESR2	Estrogen receptor 2
DPP4	Dipeptidyl peptidase 4
MAPK14	Mitogen-activated protein kinase 14
GSK3B	Glycogen synthase kinase 3 beta
HSP90AA1	Heat shock protein 90 alpha family class A member 1
MAOB	Monoamine oxidase B
ACHE	Acetylcholinesterase (Cartwright blood group)
JUN	Jun protooncogene, AP-1 transcription factor subunit
IL4	Interleukin 4
SIRT1	Sirtuin 1
CHRM3	Cholinergic receptor muscarinic 3
KCNH2	Potassium voltage-gated channel subfamily H member 2
SCN5A	Sodium voltage-gated channel alpha subunit 5
HTR3A	5-Hydroxytryptamine receptor 3A
ADRA1B	Adrenoceptor alpha 1B
NCOA2	Nuclear receptor coactivator 2
DRD1	Dopamine receptor D1
CHRM4	Cholinergic receptor muscarinic 4
HTR2A	5-Hydroxytryptamine receptor 2A
CHRM2	Cholinergic receptor muscarinic 2
CHRNA2	Cholinergic receptor nicotinic alpha 2 subunit
OPRM1	Opioid receptor Mu 1
GABRA1	Gamma-aminobutyric acid type A receptor subunit alpha1
BCL2	BCL2 apoptosis regulator
BAX	BCL2-associated X, apoptosis regulator
CASP9	Caspase-9
CASP3	Caspase-3
TGFB1	Transforming growth factor beta 1
PON1	Paraoxonase 1
MAP2	Microtubule-associated protein 2
GRIA2	Glutamate ionotropic receptor AMPA type subunit 2
NCOA1	Nuclear receptor coactivator 1
STAT3	Signal transducer and activator of transcription 3
AKT1	AKT serine/threonine kinase 1
VEGFA	Vascular endothelial growth factor A
FOS	Fos protooncogene, AP-1 transcription factor subunit
CD40LG	CD40 ligand
NFKBIA	NFKB inhibitor alpha
SOD1	Superoxide dismutase 1
HIF1A	Hypoxia-inducible factor 1 subunit alpha
FAS	Fas cell surface death receptor
VCAM1	Vascular cell adhesion molecule 1
PLAT	Plasminogen activator, tissue type
CYP19A1	Cytochrome P450 family 19 subfamily A member 1
GSTP1	Glutathione S-transferase Pi 1
SELP	Selectin P
AGTR1	Angiotensin II receptor type 1
AKR1B1	Aldo-keto reductase family 1 member B
IFNB1	Interferon beta 1
GPT	Glutamic--pyruvic transaminase
PGP	Phosphoglycolate phosphatase
IFNA1	Interferon alpha 1
LEPR	Leptin receptor
F2R	Coagulation factor II thrombin receptor

The article "Screening and Identification of Antidepressant Active Ingredients from Puerariae Radix Extract and Study on Its Mechanism" was retracted in 2024. Reasons: signs of a paper mill; suspected computer-generated content; unreliable results or conclusions; concerns about the data.

**Table 3:** Core antidepressant targets of *Puerariae Radix* and their topological characteristics.

Core gene	Target name	Degree	Betweenness centrality
AKT1	AKT serine/threonine kinase 1	33	0.1808849
FOS	Fos protooncogene, AP-1 transcription factor subunit	28	0.12839175
CASP3	Caspase-3	27	0.05017522
JUN	Jun protooncogene, AP-1 transcription factor subunit	25	0.04969618
VEGFA	Vascular endothelial growth factor A	25	0.0346735
STAT3	Signal transducer and activator of transcription 3	24	0.02416106
PTGS2	Prostaglandin-endoperoxide synthase 2	22	0.01342578
MAPK14	Mitogen-activated protein kinase 14	20	0.00748504
ESR1	Estrogen receptor 1	19	0.00626354
SIRT1	Sirtuin 1	19	0.01170971
HSP90AA1	Heat shock protein 90 alpha family class A member	18	0.04733413
ACHE	Acetylcholinesterase (cartwright blood group)	18	0.07253423
SOD1	Superoxide dismutase 1, soluble	17	0.02514393
HIF1A	Hypoxia-inducible factor 1 alpha subunit	17	0.00556528
AR	Androgen receptor	16	0.0133448

## Data Availability

The raw data supporting the conclusions of this article will be made available by the authors, without undue reservation.

The article "Screening and Identification of Antidepressant Active Ingredients from Puerariae Radix Extract and Study on Its Mechanism" was retracted in 2024. Reasons: signs of a paper mill; suspected computer-generated content; unreliable results or conclusions; concerns about the data.

## References

[1] LeMoult J., Gotlib I. H. (2019). Depression: a cognitive perspective. *Clinical Psychology Review*.

[2] Thapar A., Collishaw S., Pine D. S. (2012). Depression in adolescence. *The Lancet*.

[3] Lim G. Y., Tam W. W., Lu Y., Ho C. S., Zhang M. W., Ho R. C. (2018). Prevalence of depression in the community from 30 countries between 1994 and 2014. *Scientific Reports*.

[4] Avenevoli S., Swendsen J., He J. P., Burstein M., Merikangas K. R. (2015). Major depression in the national comorbidity survey-adolescent supplement: prevalence, correlates, and treatment. *Journal of the American Academy of Child and Adolescent Psychiatry*.

[5] Ruckenstein M. (2019). Tracing medicinal agencies: antidepressants and life-effects. *Social Science & Medicine*.

[6] Wang Y. S., Shen C. Y., Jiang J. G. (2019). Antidepressant active ingredients from herbs and nutraceuticals used in TCM: pharmacological mechanisms and prospects for drug discovery. *Pharmacological Research*.

[7] Editorial commission of Traditional Chinese Medicine (2015). State Administration of Traditional Chinese Medicine. *Traditional Chinese Medicine*.

[8] Song W., Li Y. J., Qiao X., Qian Y., Ye M. (2014). Chemistry of the Chinese herbal medicine Puerariae Radix (Ge-Gen): a review. *Journal of Chinese Pharmaceutical Sciences*.

[9] Wenli Y., Yaping Z., Bo S. (2004). The radical scavenging activities of _radix puerariae_ isoflavonoids: A chemiluminescence study. *Food Chemistry*.

[10] Zhou X., Lam W. P., Tang H. C. (2016). Effects of Gegen (_Puerariae lobatae_ Radix) water extract on improving detrusor overactivity in spontaneously hypertensive rats. *Phytomedicine*.

[11] Chen C. H., Wu S. H., Tseng Y. M. (2017). Suppressive effects of Puerariae Radix on the breast tumor incidence in rats treated with DMBA. *The Journal of Agricultural Science*.

[12] Shukla R., Banerjee S., Tripathi Y. B. (2018). Antioxidant and antiapoptotic effect of aqueous extract of Pueraria tuberosa (Roxb. Ex Willd.) DC. On streptozotocin-induced diabetic nephropathy in rats. *BMC Complementary and Alternative Medicine*.

[13] Zhang D., Ma G., Hou M., Zhang T., Chen L., Zhao C. (2016). The neuroprotective effect of puerarin in acute spinal cord injury rats. *Cellular Physiology and Biochemistry*.

[14] Yan B., Wang D., Xing D. (2004). The antidepressant effect of ethanol extract of Radix Puerariae in mice exposed to cerebral ischemia reperfusion. *Pharmacology, Biochemistry, and Behavior*.

[15] Kang E. Y., Kim H. K., Jung J. Y. (2021). Combined extract of Leonurus japonicus Houtt, Eclipta prostrata L., and Pueraria lobata Ohwi improved hot flashes and depression in an ovariectomized rat model of menopause. *Food*.

The article "Screening and Identification of Antidepressant Active Ingredients from Puerariae Radix Extract and Study on Its Mechanism" was retracted in 2024. Reasons: signs of a paper mill; suspected computer-generated content; unreliable results or conclusions; concerns about the data.

[16] Luo C., Ke Y., Yuan Y. (2016). A novel herbal treatment reduces depressive-like behaviors and increases brain-derived neurotrophic factor levels in the brain of type 2 diabetic rats. *Neuropsychiatric Disease and Treatment*.

[17] Lan J., Yan B., Zhao Y.'. (2008). Cerebral ischemia reperfusion exacerbates and pueraria flavonoids attenuate depressive responses to stress in mice. *Tsinghua Sci Technol 2008*.

[18] Li Y. H., Zhang C. H., Qiu J. (2014). Antidepressant-like effects of Chaihu-Shugan-San via SAPK/JNK signal transduction in rat models of depression. *Pharmacognosy Magazine*.

[19] Mahdy H. M., Mohamed M. R., Emam M. A., Karim A. M., Abdel-Naim A. B., Khalifa A. E. (2014). Puerarin ameliorates 3-nitropropionic acid-induced neurotoxicity in rats: possible neuromodulation and antioxidant mechanisms. *Neurochemical Research*.

[20] Zhao Y., Hu B., Liu Q., Wang Y., Zhao Y., Zhu X. (2021). Social support and sleep quality in patients with stroke: the mediating roles of depression and anxiety symptoms. *International Journal of Nursing Practice*.

[21] Tian W., Zhao J., Lee J. H. (2020). Neuroprotective effects of Cornus officinalis on stress-induced hippocampal deficits in rats and H_2_O_2_-induced neurotoxicity in SH-SY5Y neuroblastoma cells. *Antioxidants*.

[22] Sun L., Ye R., Liang R., Xing F. (2020). Treadmill running attenuates neonatal hypoxia induced adult depressive symptoms and promoted hippocampal neural stem cell differentiation via modulating AMPK-mediated mitochondrial functions. *Biochemical and Biophysical Research Communications*.

[23] Arioz B. I., Tastan B., Tarakcioglu E. (2019). Melatonin attenuates LPS-induced acute depressive-like behaviors and microglial NLRP3 inflammasome activation through the SIRT1/Nrf2 pathway. *Frontiers in Immunology*.

[24] Liu X. J., Li Z. Y., Li Z. F. (2012). Urinary metabonomic study using a CUMS rat model of depression. *Magnetic Resonance in Chemistry*.

[25] Zhang L., Zhu Z., Tan Z., Luo H., Hu X., Li Y. (2017). Docosahexaenoic acid induces glial cell-line derived neurotrophic factor release in C6 glioma cells: implications of antidepressant effects for docosahexaenoic acid. *Biochemical and Biophysical Research Communications*.

[26] Liu Y., Shen S., Li Z. (2014). Cajaninstilbene acid protects corticosterone-induced injury in PC12 cells by inhibiting oxidative and endoplasmic reticulum stress-mediated apoptosis. *Neurochemistry International*.

[27] Nissanka N., Moraes C. T. (2018). Mitochondrial DNA damage and reactive oxygen species in neurodegenerative disease. *FEBS Letters*.

The article "Screening and Identification of Antidepressant Active Ingredients from Puerariae Radix Extract and Study on Its Mechanism" was retracted in 2024. Reasons: signs of a paper mill; suspected computer-generated content; unreliable results or conclusions; concerns about the data.

[28] Yamada J., Jinno S. (2016). Aging of hippocampal neurogenesis and soy isoflavone. *Oncotarget*.

[29] Zakeri M., Monajjemi M. (2018). Effective molecules of some natural product as antidepressant and antihistamine drugs: A NMR study. *Ukrainian Journal of Ecology*.

[30] Tian Z., Liu S., Wang Y., Li X. Q., Zheng L. H., Zhao M. G. (2013). Neuroprotective effects of formononetin against NMDA-induced apoptosis in cortical neurons. *Phytotherapy Research*.

[31] Wen X. D., Qi L. W., Li B. (2009). Microsomal metabolism of calycosin, formononetin and drug-drug interactions by dynamic microdialysis sampling and HPLC-DAD-MS analysis. *Journal of Pharmaceutical and Biomedical Analysis*.

[32] Qiu Z. K., Zhang G. H., Zhong D. S. (2017). Puerarin ameliorated the behavioral deficits induced by chronic stress in rats. *Scientific Reports*.

[33] Cheng J., Chen M., Zhu J. X. (2019). FGF-2 signaling activation in the hippocampus contributes to the behavioral and cellular responses to puerarin. *Biochemical Pharmacology*.

[34] Zhao J., Luo D., Liang Z., Lao L., Rong J. (2017). Plant natural product puerarin ameliorates depressive behaviors and chronic pain in mice with spared nerve injury (SNI). *Molecular Neurobiology*.

[35] Losenkov I. S., Vyalova N. M., Simutkin G. G., Bokhan N. A., Ivanova S. A. (2016). An association of AKT1 gene polymorphism with antidepressant treatment response. *The World Journal of Biological Psychiatry*.

[36] Kemp A., Tischmeyer W., Manahan-Vaughan D. (2013). Learning-facilitated long-term depression requires activation of the immediate early gene, c-fos, and is transcription dependent. *Behavioural Brain Research*.

[37] Gałecki P., Gałecka E., Maes M. (2013). Vascular endothelial growth factor gene (_VEGFA_) polymorphisms may serve as prognostic factors for recurrent depressive disorder development. *Progress in Neuro-Psychopharmacology and Biological Psychiatry*.

[38] Kwon S. H., Han J. K., Choi M. (2017). Dysfunction of Microglial STAT3 Alleviates Depressive Behavior via Neuron- Microglia Interactions. *Neuropsychopharmacology*.

[39] Labaka A., Gómez-Lázaro E., Vegas O., Pérez-Tejada J., Arregi A., Garmendia L. (2017). Reduced hippocampal IL-10 expression, altered monoaminergic activity and anxiety and depressive-like behavior in female mice subjected to chronic social instability stress. *Behavioural Brain Research*.

[40] Nowacka M. M., Obuchowicz E. (2012). Vascular endothelial growth factor (VEGF) and its role in the central nervous system: a new element in the neurotrophic hypothesis of antidepressant drug action. *Neuropeptides*.

[41] Shibata T., Yamagata H., Uchida S. (2013). The alteration of hypoxia inducible factor-1 (HIF-1) and its target genes in mood disorder patients. *Progress in Neuro-Psychopharmacology and Biological Psychiatry*.

The article "Screening and Identification of Antidepressant Active Ingredients from Puerariae Radix Extract and Study on Its Mechanism" was retracted in 2024. Reasons: signs of a paper mill; suspected computer-generated content; unreliable results or conclusions; concerns about the data.

[42] Milaneschi Y., Lamers F., Berk M., Penninx B. W. J. H. (2020). Depression heterogeneity and its biological underpinnings: toward immunometabolic depression. *Biological Psychiatry*.

